# A Narrative Review of the Antitumor Activity of Monoterpenes from Essential Oils: An Update

**DOI:** 10.1155/2022/6317201

**Published:** 2022-05-24

**Authors:** Thaíssa Q. Machado, Anna C. C. da Fonseca, Allana B. S. Duarte, Bruno K. Robbs, Damião P. de Sousa

**Affiliations:** ^1^Postgraduate Program in Applied Science for Health Products, Faculty of Pharmacy, Fluminense Federal University (UFF), CEP: 24010-141 Niteroi, Brazil; ^2^Postgraduate Program in Dentistry, Health Institute of Nova Friburgo (ISNF), Fluminense Federal University (UFF), CEP: 28625-650 Nova Friburgo, RJ, Brazil; ^3^Postgraduate Program in Natural and Synthetic Bioactive Products, Federal University of Paraíba, 58051-970 João Pessoa, PB, Brazil; ^4^Basic Science Department, ISNF/UFF, CEP: 28625-650 Nova Friburgo, RJ, Brazil; ^5^Department of Pharmaceutical Sciences, Federal University of Paraíba, 58051-970 João Pessoa, PB, Brazil

## Abstract

Monoterpenes are a group of natural products that have been widely studied due to their therapeutic potential against various pathologies. These compounds are abundant in the chemical composition of essential oils. Cancer is a term that covers more than 100 different types of malignant diseases and is among the leading causes of death in the world. Therefore, the search for new pharmacotherapeutic options applicable to cancer is urgent. In this review, studies on the antitumor activity of monoterpenes found in essential oils were selected, and botanical, chemical, and pharmacological aspects were discussed. The most investigated monoterpenes were carvacrol and linalool with highly significant *in vitro* and *in vivo* tumor inhibition in several types of cancers. The action mechanisms of these natural products are also presented and are wildly varied being apoptosis the most prevalent followed by cell cycle impairment, ROS production, autophagy, necroptosis, and others. The studies reported here confirm the antitumor properties of monoterpenes and their anticancer potential against various types of tumors, as demonstrated in *in vitro* and *in vivo* studies using various types of cancer cells and tumors in animal models. The data described serve as a reference for the advancement in the mechanistic studies of these compounds and in the preparation of synthetic derivatives or analogues with a better antitumor profile.

## 1. Introduction

Cancer is a leading cause of death worldwide and so an important public health issue. Aging, population growth, and risk factors related to socioeconomic development are the main causes of cancer boost. In 2020, it was estimated that there were 19.3 million new cancer cases and nearly 10.0 million cancer deaths, with female breast, lung, colorectal, prostate, and stomach cancers topping the incidence list [1]. Chemotherapy represents the main conduct in the treatment of cancer. However, many chemotherapeutics not only kill cancer cells but also affect normal cells and tissues, which demonstrate a need to search for more selective active compounds that develop fewer side effects [2, 3].

Several drugs used in cancer treatment are natural products or derivatives of them, such as taxol, isolated from *Taxus baccata* and the analogs docetaxel (Taxotere) and cabazitaxel (Jevtana) in addition to vincristine and vinblastine (Velban) derived from *Catharanthus roseus* and their analogues vindesine (Eldisine) and vinorelbine (Navelbine) [3, 4]. In addition, of 175 molecules approved for antitumor therapy between 1940 and 2014, approximately 50% were derived from natural products or their derivatives [5, 6]. Thus, natural products represent a significant source of antitumor agents whose pharmacological action and clinical application has demonstrated success in cancer therapy [2]. The mixture of volatile compounds from plants known as essential oil plays a significant role in plant defense. The oil is made up of hundreds of compounds that are mainly represented by terpenoids. Essential oils have antitumor activity against several types of tumors, such as hepatocellular carcinoma, triple negative breast cancer, and acute myeloid leukemia (AML), in addition to presenting low toxicity [7–11]. The essential oil of leaves from *Zornia brasiliensis* and *Guatteria friesiana* (W. A. Rodrigues), plants used in folk medicine in Brazil and Colombia, have terpenoids as its main components and are highly cytotoxic and inhibit tumor growth from several types of cancer both *in vitro* and *in vivo* [12, 13]. The anticancer potential of monoterpenes found in essential oils has also been reported [7, 14]. Essential oil from the leaves of *Croton regelianus* Muell. Arg., a native plant from Northeast Brazil used in folk medicine, has ascaridole, a monoterpene, as one of the main constituents with high antitumor activity against leukemia, glioblastoma, and sarcomas in mice models [15]. Furthermore, monoterpenes (-)-*α*-pinene, (-)-*β*-pinene, and limonene from essential oils from *Piper rivinoides* Kunth were active against tumor cell lines of oral squamous cell carcinoma (SCC9 and SCC25), showing greater selectivity in relation to carboplatin, the drug of choice in the clinic [16]. Thus, as described in Method, the present study performed an up-to-date review of essential oil monoterpenes with antitumor activity.

## 2. Method

The present review was based in data search performed in the scientific literature database PubMed, the most accessed for biomedical (medicine and health) literature worldwide. The eligibility criteria and selection of the studies were based on the following keywords: monoterpene, essential oils, antitumoral, anticancer, and cytotoxicity, and covered a period from January 2014 to December 2020, that way, performing an update on our previous review published in 2014 [14]. The scientific publications were selected from studies published in English and discussed in this manuscript.

## 3. Results and Discussion

This discussion focused on the *in vitro* and *in vivo* antitumoral role of essential oil monoterpenes was based on studies indexed in the biomedical database PubMed and as described in Method.

Chemical structures and names of antitumor monoterpenes are provided in Figure 1.

### 3.1. Monoterpenes That Induced Apoptosis as a Pathway of Death

#### 3.1.1. 1,8-Cineole

1,8-Cineole demonstrated promising cytotoxic and proapoptotic properties, which showed cytotoxicity against A2780 cells comparable with that of doxorubicin, enhanced apoptosis in A2780 cell, and caused a dose-dependent increase in preG1 cell cycle events [17]. Furthermore, 1,8-cineole induced the apoptosis and G2/M phase arrest of cell cycle in A431 cells by increasing the expression of p53. Also, there was the expression of apoptotic proteins, such as Bax/Bcl-2, Cyt-c, caspase-9, and caspase-3. Molecular docking simulations predicted the hydrophobic interaction between 1,8-cineole with PARP1 receptor and Bcl-2 [18]. 1,8-Cineole was selective, and it did not affect cell viability of normal lung WI-38 cells and inhibited A549 cell migration but did not induce apoptosis [19].

#### 3.1.2. *α*-Thujone

*α*-Thujone has demonstrated several pharmacological effects, such as antitumor, analgesic, and insecticide. It was seen that *α*-thujone has not shown cytotoxicity to HCT116 and SW620 cells; however, it increased the proliferation of CD3AK immune cells and its cytotoxicity against cancer cells by improving the expression of CD107a, p-Akt, and p-ERK1/2 [20]. Furthermore, *α*-thujone also exerted effect on GBM (glioblastoma) cells. The observed effects were induction of apoptosis, considerable inhibition of cell motility, induction of oxidative stress, and autophagy in *α*-thujone-treated tumor cells. Meanwhile, normal astrocytes showed lower sensitivity to *α*-thujone treatment [21].

#### 3.1.3. Bornyl Acetate

The combination of bornyl acetate with 5-fluorouracil potentiated the anticancer activity of 5-fluorouracil in human gastric cancer (SGC-7901) cells. The results of this combination were induction of apoptosis, DNA fragmentation, G2/M cell cycle arrest, cell morphology alterations, and potentiated effect of cell growth inhibition, indicating a synergistic enhancement in the anticancer activity of 5-fluorouracil [22].

#### 3.1.4. *β*-Pinene

(-)-*β*-Pinene has demonstrated a cytotoxic effect against tumor cells. It was observed in human oral tongue cancer cells that (-)-*β*-pinene showed cytotoxicity, altered cell morphology, large amounts of pyknotic nuclei, membrane blebs, and cell shrinkage, and caspase inhibitors ZVAD (pancaspase) and ZDEVD (caspase-3) reduced cell death. In addition, (-)-*β*-pinene also showed selectivity in primary normal human gingival fibroblast [16]. *β*-Pinene has also been evaluated in association with an already established drug, paclitaxel, in non-small-cell lung cancer cells. The results revealed that the combination of paclitaxel with *β*-pinene showed a substantial synergistic effect. Furthermore, paclitaxel+*β*-pinene showed morphological change characteristic of apoptosis like chromatin condensation and fragmentation of the nucleus [23].

#### 3.1.5. Carvone

Carvone is a monocyclic monoterpene that has been reported to have antioxidant, antimicrobial, anticonvulsant, and antitumor activities. Regarding the antioxidant effect, it was seen that carvone treatment increased levels of total antioxidant capacity in cultured primary rat neuron cells. In addition, it increased levels of total oxidative stress in primary rat neuron cultures and rat brain NB cell line N2a. There was also a reduction in cell viability rates in both cell types [24].

In addition to the antioxidant effect, carvone also showed antitumor activities. Carvone inhibited proliferation of MCF 7 and MDA MB 231 cells and inhibited the migration of these breast cancer cells. In addition, it induced apoptosis, as was seen by the fragmentation of nuclei and the presence of apoptotic bodies, and it also arrested MCF 7 cells in the S phase of the cell cycle, caused DNA damage and ROS production, and increased levels of p53, Bad, cleaved caspase-3, and cleaved PARP [25]. Carvone also exerted anticancer effects on myeloma cancer cells (KMS-5) with antiproliferative effects that were associated with the induction of apoptosis and arrest of the G2/M cell cycle. It has also been seen that carvone can inhibit cell invasion and protein expression p-P38 at IC50 [26]. Another effect observed was with carvone associated with doxorubicin, in which carvone showed a synergistic anticancer effect with doxorubicin on the MCF 7 cell line, in addition to decreasing the toxicity of doxorubicin on a normal heart cell line. In BALB/c mice, carvone protected the heart from doxorubicin toxicity. The protective effect of carvone was due to an increase in catalase activity [27]. Carvone also prevented skin carcinogenesis and reduced levels of phase I enzymes (Cyt P450 e-Cyt b5) with increased levels of phase II enzymes (GR, GST, and GSH). There was also increase in the expression of Bax, caspase-3, and caspase-9 with decreased expression of mutated p53 and Bcl-2 in Swiss albino mice treated with DMBA (7, 12-dimethylbenz [a] anthracene) and D-carvone [28].

#### 3.1.6. Limonene

Limonene effects have recently been investigated on T24 human bladder cancer cells presenting an IC50 of 9 *μ*M. Ye et al. demonstrated that it presented the antitumor capacity to induce cell cycle arrest, suppression of cell migration and invasion, and apoptosis with observation of nuclear fragmentation, chromatin condensation, splitting of the nucleus, increase of Bax and caspase-3, and decrease of Bcl-2 expressions [29]. D-limonene showed lung antitumor activity *in vivo* and *in vitro* by preventing the growth of lung cancer cells and inducing apoptosis through mechanisms involving autophagy. There was an increase in Bax and cleaved PARP during treatment, which may be related to induce death of lung cancer cells. Increases were also found in Atg-5, presuming that Atg5 overload may be partially involved in D-limonene-induced apoptosis [30].

#### 3.1.7. Thymoquinone

It has recently been demonstrated that thymoquinone induces apoptosis of 786-O human renal carcinoma cells. In more details, it decreases cell viability in a concentration- and time-dependent manner with an IC50 of 3.8–12.9 *μ*M, increases intracellular ROS levels and the sub-G1 population, and decreases the migration and invasiveness potential of tumor cells [31]. Thymoquinone reduced viability and increased cell death due to apoptosis in human lung tumor cells A549 presenting the highest IC50 against cancer cells at 47 ± 0.09 *μ*M. The approach with this monoterpene significantly increased the Bax/Bcl-2 ratio, positively regulated the expression of p53, and activated caspase-dependent apoptosis by the activation of caspases-3 and -9 [32].

### 3.2. Monoterpenes That Induced Apoptosis and Tumor Inhibition *In Vivo*

#### 3.2.1. *α*-Pinene

The *α*-pinene is a natural compound that has demonstrated anticancer activity. The *α*-pinene inhibited liver cancer cell growth. In nude mice with hepatocellular carcinoma, Chk1 and Chk2 levels were upregulated, Cyclin B, CDC25, and CDK1 levels were downregulated, and the average tumor size was significantly smaller in mice treated with *α*-pinene. The average tumor was significantly lighter than the control, and histology examination of xenografts showed more slow-growing cells and dead cells. *α*-Pinene also caused marked accumulation of a G2/M population in BEL-7402 cells [19]. In human cancer ovary (PA-1) cells, *α*-pinene inhibited the cycle progression at G2 to M phase and markedly increased caspase-3-dependent apoptotic cell death [33]. It was also observed that HepG2 cells treated with *α*-pinene exhibited growth inhibition, G2/M-phase cell cycle arrest, triggered oxidative stress, and induced apoptosis. The cell cycle arrest was associated with downregulated cyclin-dependent kinase 1 (CDK1) and miR-221 levels. There were also upregulated levels of CDKN1B/p27, *γ*-H2AX, phosphorylated ATM, phosphorylated Chk2, and phosphorylated p53 [34]. The combination of paclitaxel with *α*-pinene showed a substantial synergistic effect, showing consequences on cell cycle distributions of A549 cells, in which the percentage of sub-G0/G1-phase cells was decreased on the addition of *α*-pinene to paclitaxel, and the population of G0/G1 cells was increased presenting morphological change characteristic of apoptosis [23]. *α*-Pinene also demonstrated protective effect against ultraviolet A-induced cellular damages in human skin epidermal keratinocytes (HaCaT cells). *α*-Pinene showed a probable antioxidant property, preventing UVA-induced cytotoxicity, generation of ROS, lipid peroxidation, and DNA stand breaks. Furthermore, *α*-pinene inhibited inflammatory mediators such as NF-*κ*B, TNF-*α*, and IL-6 expression and also modulated nucleotide excision repair proteins via activation of p53 and p21 that prevent the formation of UVA-induced cyclobutane pyrimidine dimers [35].

#### 3.2.2. Borneol

Natural borneol (NB) has been used as a promoter of drug absorption; thus, it was seen that borneol could potentiate the cellular uptake of bisdemethoxycurcumin (possible anticancer activity) [36]. Besides that, borneol can also act as an “upper guiding drug,” because it has a potential autophagic inhibitor activity that may guide luteolin (anticancer activity) in the ubiquitin-proteasome pathway and the ubiquitin-signal autophagic degradation [37]. It was also seen that borneol increased the blood-brain barrier permeability and intracellular uptake of doxorubicin (DOX), which potentiated DOX-induced G2/M cell cycle arrest and inhibited U251 human glioma xenograft growth *in vivo* through combined treatment of DOX with natural borneol [38]. The effect of borneol was also seen in combination with cisplatin, and it was seen that borneol synergistically enhanced the anticancer activity of cisplatin in human glioma cells. Cotreatment of cisplatin inhibited U251 cell viability and enhanced cisplatin-induced apoptosis with caspase activation and reactive oxygen species overproduction, and borneol also increased cisplatin-induced cell growth in a ROS-dependent manner [39].

#### 3.2.3. Camphene

Camphene is a bicyclic monoterpene and a component of essential oils derived from plants such as rosemary, turmeric, pine, and ginger that has high antioxidant, anti-inflammatory, and antimicrobial activity [40, 41]. The *in vitro* activity of camphene induced apoptosis by the intrinsic pathway in melanoma cells causing endoplasmic reticulum stress. Moreover, there were also release of Ca2þ together with calreticulin and HmgB1, upregulation of caspase-3 activity, and loss of mitochondrial membrane potential. Camphene was also evaluated *in vivo*, in male C57Bl/6 mice, inhibiting subcutaneous tumor growth of highly aggressive melanoma cells in a syngeneic model [42].

#### 3.2.4. Carvacrol

Carvacrol, when tested on AGS (human gastric adenocarcinomas) and WS-1 (normal human fibroblastic cells), had toxic effects but was more effective in cancer cells. One possible mechanism was apoptosis induced by DNA damage [43]. Carvacrol also induced apoptosis in different cells, such as A549 cells, DU145, human colon cancer cell lines, HL-60, Jurkat, and PC-3 [44–48]. Apoptosis occurred in A549 cells through activation of key regulators of apoptosis, such as p-JNK and Bax, and reduction of Bcl2, release of cytochrome C, activation of the caspase cascade, and production of reactive oxygen species (ROS) [44]. In DU145, apoptosis occurred with increased generation of ROS, disruption in the mitochondrial membrane potential, and arrest in the G0/G1 phase of the cell cycle [45]. In human colon cancer cell lines, there was also cell apoptosis with cell cycle arrest in the G2/M phase, decrease in expression of cyclin B1, downregulation in the expression of Bcl-2, induction in the phosphorylation of extracellular regulated protein kinase and protein kinase B (p-Akt), and upregulation in the expression of Bax N-terminal kinase and c-Jun [46]. In HL-60 (human acute promyelocytic leukemia cells) and Jurkat (human T lymphocyte cells), apoptosis occurred with the formation of free radicals, reduced levels of antioxidants such as catalase and superoxide dismutase, increased Bax expression, and decreased Bcl-2 expression, and apoptosis by carvacrol was mediated by caspase-3 [47]. In addition, apoptosis acted in reducing the cell viability of PC-3 cells (prostate cancer cell line), showing high levels of ROS, disruption of the mitochondrial membrane potential, prevented cell cycle in G0/G1, decline in the expression of cyclin D1 and cyclin-dependent kinase 4 (CDK4), and increased expression of the CDK inhibitor p21 [48].

Cisplatin (CP) and carvacrol showed dose-dependent cytotoxicity and activated ERK1/2. The MEK inhibitor PD325901 suppressed ERK expression, increased cytotoxicity of carvacrol, increased viability of cells by modulating apoptosis, and increased microtubule-associated protein 1A/1B-light chain 3 beta expression in cisplatin treatment. Cotreatment with cisplatin and carvacrol increased the viability of cancer cells compared to treatment with CP, due to the suppression of apoptosis. MEK inhibition decreased cell viability, without causing changes in apoptosis. The carvacrol also increased cisplatin-induced expression of light chain 3 beta. It induced CP resistance in HeLa cells through ERK1/2-independent suppression of apoptosis and ERK1/2-dependent modulation of autophagy [49].

Other effects were observed, as alteration of soluble factors in HCT-116 and HT-29 (human colorectal carcinoma) [50]. Carvacrol also suppressed cell proliferation and migration, and its inhibitory effect was attenuated in NSCLC (non-small-cell lung cancer) cells with overexpression of AXL, in which the treatment promoted downregulation of AXL expression and inhibited AXL phosphorylation after ligand stimulation [51]. It was able to inhibit cell proliferation, prevent metastasis in hepatocellular carcinogenesis, and suppress the elevation of serum tumor marker enzymes, carcinoembryonic antigen, and alpha-feto protein induced by diethylnitrosamine [52]. It did not show mutagenic effects on human lymphocytes but showed that at concentrations above 100 mg/L there was a decrease in cell viability. Furthermore, it caused statistically significant increases in the levels of TAC (total antioxidant capacity) and TOS (total oxidative stress) on human lymphocytes [53]. *In vivo*, changes in body weight and oxidative stress index were found in plasma and stomach tissues of treated Wistar rats [43].

#### 3.2.5. Citral

Citral had an antiproliferative effect on several cancer cells. Apoptosis was observed in human stomach cancer cells [54]; in prostate cancer cells (PC3 cells) through upregulating BAX and downregulating Bcl-2 expression [55]; and in HCT116 and HT29 (colorectal cancer cell lines), in which it induced mitochondrial-mediated apoptosis via increased intracellular ROS and phosphorylation of p53 protein and the expression of Bax and decreased expression of Bcl-2 and Bcl-xL which promoted the cleavage of caspase-3 [56]; and citral also showed cytotoxicity in Burkitt's lymphoma cell line human and additively increased the cytotoxic and apoptotic effects of doxorubicin [57]. The combination of citral and doxorubicin increased the expression of the proapoptotic protein BAK but decreased the expression of the antiapoptotic protein BCL-XL compared to cells just treated with doxorubicin [57].

In addition to apoptosis, citral also induced cytotoxicity by regulating several genes involved in signaling pathways, inhibiting metastases, inhibiting colony formation, and interrupting migration of colonies of cancer cells [54]. Furthermore, it was able to block the growth of breast tumor mediated by ALDH1A3 through its inhibition. Inhibition of ALDH1A3 blocked the colony formation and activity regulating gene expression [58]. Other effects caused by citral were the damage to the clonogenic property and changes in morphology of cancer cells and suppression of lipogenesis of prostate cancer cells [54].

Studies also have suggested that citral binds to MARK4, inhibiting its enzyme activity, which is associated with the cell cycle and, therefore, cancer. Moreover, it also inhibited proliferation of the breast cancer cell line MCF-7 [59]. It was also seen that treatment with citral reduced the size and number of cells with ALDH+ activity of the tumors in BALB/c mice challenged with 4T1. Furthermore, smaller tumors and delayed tumorigenicity were observed in mice treated with citral after undergoing primary tumor cell reimplantation [60].

#### 3.2.6. Citronellol

Citronellol has been described with antitumor activity against lung [61] and breast cancers [62], inducing necroptosis and apoptosis, respectively. For lung cancer, IC50 was found to be 49.74 *μ*g/mL and necroptosis was confirmed by an upregulation of TNF-*α* pathway and downregulation of caspase-3 and -8 activities. Besides, citronellol at a dose of 50 mg/kg inhibited 80% of subcutaneous tumor growth previously induced by intraperitoneal injection of NCI-H1299 in nude mice. For breast cancer, IC50 was found to be 35 and 80 *μ*M, using two different tumor cell lines, and apoptosis was validated by the loss of cell viability, increase in ROS generation, altered mitochondrial membrane potential, enhanced DNA damage, and modulation of the expression of apoptotic proteins (inhibition of Bcl-2 with upregulation of Bax and caspase-9 and -7) in MCF-7 and MDA-MB-231 cells.

#### 3.2.7. Geraniol and Geranyl Acetate

Qi et al. showed that geraniol and geranyl acetate induce apoptosis with upregulation of Bax and downregulation of Bcl-2 expressions, DNA damage, and cell cycle arrest on Colo-205 colon cancer cells, presenting an IC50 of 20 and 30 *μ*M [63]. However, geraniol presents antitumor activity by several other mechanisms, as observed in the past years. In an oral carcinogenesis model using a 200 mg/kg dose, geraniol downregulates the activation of NF-*κ*B, reducing the expression of TNF-*α*, IL-1*β*, COX-2, and iNOS [64]. On PC-3 prostate cancer cells, using microarray, it was observed that geraniol downregulates the transcription factor E2F8 suppressing cell growth and inducing G2/M arrest [65]. On lung adenocarcinoma cancer cells, with an IC50 of 797.2 *μ*M and *in vivo* doses of 50 and 75 mmol G/kg, it inhibits the mevalonate pathway resulting in growth inhibition of A549 cells and *in vivo* subcutaneous tumor growth besides promotion of apoptosis [66]. On Ishikawa endometrial cancer cells, with an IC50 of 140.929 *μ*M, geraniol induces apoptosis with the involvement of the mitochondrial pathway, observed by a decrease in Bcl-2 and increase in Bax staining and TUNEL-positive cells, as well as an increase in the mRNA levels of Bax, caspase-3 and -8, cytochrome C, and Fas and a decrease in the Bcl-2 gene [67].

#### 3.2.8. Linalool

Linalool has been a major topic of investigation over the last years. Its acts against several types of cancer mainly through induction of cell cycle arrest and oxidative stress. On A549 lung adenocarcinoma cells, linalool suppresses cell growth through cell cycle arrest, and oxidative stress also acts on the mitochondrial membrane potential depolarization and inhibition of cell proliferation, besides preventing cell migration [19]. On OECM 1 oral cancer cells, with an IC50 of 10 *μ*M, it inhibits the viability of cells and induces cell cycle arrest and apoptosis with a decrease in the expression of p-PI3K, p-AKT, and Bcl-2 and a rise in the expression of Bax [68]. On HCT 116 colon cancer cells, linalool promotes apoptosis via lipid peroxidation observed *in vitro* and *in vivo*; moreover, it induces a reduction of 55% in mean xenograft subcutaneous tumor weight in a 200 mg/kg dose [69]. On T-47D breast, SW 620 colorectal and HepG2 liver cancer cells, with IC50 of 224, 222, and 290 *μ*M, linalool induced a concentration of cells in the G1 phase and by cytokine array analysis observed a stimulation of IFN-*γ*, IL-13, IL-2, IL-21, IL-21R, IL-4, IL-6sR, and TNF-*α* secretion, suggesting it could also induce Th1 cellular immune response [70]. On HepG2 hepatocellular carcinoma cells, it induces cell cycle arrest and apoptosis with the involvement of Ras, MAPKs, and Akt/mTOR pathways, besides ROS production influencing cytotoxicity [71]. On U937 leukemia and HeLa cervical cancer cells, with an IC50 of 2.59 and 11.02 *μ*M, linalool induces cell cycle arrest facilitating the expression of p53, p21, p27, p16, and p18 [72]. On sarcoma-180 cells *in vitro* and in a solid tumor model, linalool appeared to be selectively cytotoxic towards tumor cells in contrast to conventional chemotherapeutic drug, presenting reduction in cell viability, tumor volume, tumor weight, and tumor cell count data; furthermore, it induces apoptosis and cell cycle arrest in tumor cells and extensive necrosis and reduced viable tissue mass *in vivo* [73].

#### 3.2.9. Perillyl Alcohol, Perillaldehyde 8,9-Epoxide, and Dehydroperillic Acid

Perillyl alcohol, its derivative (perillaldehyde 8,9-epoxide), and biotransformation metabolite (dehydroperillic acid) act against cancer in different ways. Perillyl alcohol presents an IC50 of 1.8 and 2 mM on U87 and U251 glioblastoma cells and an apoptosis induction through a signaling mechanism mediated by Na/K-ATPase [74]. Also, it has an antitumor activity by inhibiting HIF-1 in HeLa cervical, SK-Hep1 hepatic, and HCT116 colon cancer cells, which was mediated by the inhibition of the mTOR/4E-BP1 signaling pathways; moreover, in a xenograft tumor model using HCT116 cells, perillyl alcohol led to a tumor inhibition of 64.11% [75]. It was also demonstrated to induce apoptosis in an elaborated work using a chemoprevention gene therapy approach with perillyl alcohol and a replication incompetent adenovirus to deliver melanoma differentiation associated gene-7/Interleukin-24 (mda-7/IL-24) with a resulting enhanced conversion of mda-7/IL-24 mRNA into protein in AsPC-1, PANC-1, MIA PaCa-2, and BxPC-3 pancreatic cancer cells [76]. Andrade et al. showed that perillaldehyde 8,9-epoxide inhibits up to 58.7% of tumor growth in a sarcoma mouse model [77] and induces apoptosis and necrosis in OVCAR-8 ovarian, HCT-116 colon, SF-295 brain, and HL-60 leukemia tumor cells with IC50 values of 0.64-1.75 *μ*L/mg [78]. Regarding dehydroperillic acid, it was proved to inhibit DNA synthesis and promote apoptosis, being highly cytotoxic (IC50 = 125 *μ*g/mL) and selective (selective index = 400) in A549 lung cancer cells [79].

#### 3.2.10. Terpineol

Terpineol has been described as able to suppress cell migration and induce cell cycle arrest and apoptosis in HepG2 hepatic cancer cells with IC50 of 19.5 *μ*M and observation of DNA fragmentation; besides, the doses of 10 and 20 mg/kg in subcutaneous tumors promoted a reduction in the tumor weight and volume [80]. Terpineol cytotoxic role was also investigated by screening several cell lines (HT29, HCT116, COLO320, DLD1, AGS, COLO357, Panc-1, MIA-PACA, DU145, and CL-1) of colorectal, gastric, pancreatic, and prostate cancer cells showing a significant growth inhibition in all the different cancer cells. Besides inducing a decrease in subcutaneous tumor volume, importantly, it was shown to improve the effect of several anticancer agents [81]. Terpineol was also investigated on BEL-7402 liver cancer cells, presenting an IC50 of 0.32 mg/mL, inhibition of cell growth, and induction of apoptosis, with observation of cell shrinkage, deformation and vacuolization of mitochondria, nuclear chromatin condensation and fragmentation, formation of apoptotic bodies, and accumulation of cells at G1 or S phase [82].  Table 1 shows the monoterpenes and their antitumor effects on specific experimental models.

#### 3.2.11. Thymol

Thymol's antitumor activities have been largely studied over the past years. Elbe et al. have recently investigated thymol's cytotoxic effect on SKOV-3 ovarian, PC-3 and DU145 prostate, MDA-MB-231 breast, and KLN205 lung cancer cells finding IC50 values ranging from 208.36 to 799 *μ*M and apoptosis induction [83, 84]. It was also studied on T24, SW280, and J28 bladder cancer cells presenting IC50 of 90.1-130.5 *μ*M, cell cycle arrest, and mitochondria-related apoptosis with activation of the ROS-JNK/p38 pathway [85]. On Cal27, SCC4, and SCC9 oral squamous cell carcinoma cells, thymol was cytotoxic with IC50 of 300-550 *μ*M, displaying mitochondrial transmembrane potential depolarization, apoptosis, and a reduction on subcutaneous tumor volume [86]. On AGS gastric carcinoma cells, thymol inhibited cell growth and promoted apoptosis and depolarization of mitochondrial membrane potentials with morphological changes, ROS production, and activation of Bax, caspases, and PARP [87]. On A549 lung cancer cells (IC50 = 745 *μ*M), thymol induced apoptosis and cell cycle arrest with cellular and nuclear morphological changes, phosphatidylserine translocation, mitochondrial membrane depolarization, activation of caspase-3, upregulation of Bax, downregulation of Bcl-2, apoptotic fragmented DNA, and ROS production [88]. On HCT-116 colorectal carcinoma cells, thymol promoted ROS generation, induced severe damage to DNA and mitochondria, and increased the expression of PARP-1, p-JNK, cytochrome-C, and caspase-3 [89]. On MCF-7 and MDA-MB231 breast cancer cells, thymol was cytotoxic to both cell lines with IC50 of 47 and 56 *μ*g/mL and promoted ROS production mitochondrial membrane potential loss, caspase-3 activation, DNA damage, and cell cycle arrest [90]. Altogether, thymol's antineoplastic functions occur basically by induction of apoptosis and mitochondria-mediated apoptosis. Interestingly, Shettigar et al., using HepG2 hepatocarcinoma cells, have shown that thymol, at lower concentrations, can be an antioxidant and protective agent against mercuric chloride-induced deleterious effects [91], demonstrating its capacity to act not only as a prooxidant but also as an antioxidant compound, depending on its concentration. Indeed, Aydin and Türkez have also demonstrated thymol's antioxidant potential using human blood cells [92].

### 3.3. Monoterpenes That Induced Other Antitumor Mechanisms and Tumor Inhibition *In Vivo*

#### 3.3.1. Cuminaldehyde

Cuminaldehyde has been shown to possess the ability to inhibit topoisomerase I and II activities and to upregulate lysosomal vacuolation on different cancer cells, exercising antitumor activity both *in vitro* and *in vivo* [93, 94]. Using COLO 205 colorectal adenocarcinoma cells, Cherng's group found an IC50 of 16.31 *μ*M and a tumor growth inhibition of 69.4% in subcutaneous tumors with a dose of 20 mg/kg. The same group also investigated the effect of cuminaldehyde in A549 lung adenocarcinoma cells finding similar results with an IC50 of 18.33 *μ*M and a subcutaneous tumor growth inhibition of 50% using a dose of 10 or 20 mg/kg.

#### 3.3.2. Fenchone

Fenchone, a major component of *Mesosphaerum sidifolium* (Lamiaceae) oil, at a dose of 60 mg/kg, induced *in vivo* cell growth inhibition (total viable cancer cells, tumor volume, and mass) on Ehrlich ascites carcinoma model through stimulation of cell cycle arrest [95]. This bicyclic monoterpene is also present in the essential oil of fennel (*Foeniculum vulgare*) and has antioxidant, anti-inflammatory, antinociceptive, antifungal, and acaricidal properties [96, 97].

#### 3.3.3. Myrtenal

Myrtenal has been shown to cause cell death, reduce migration and invasion of B16F0, B16F10, and SkMel-5 melanoma cells *in vitro*, and significantly decrease metastasis promoted by B16F10 cells *in vivo*, using a 15 mg/kg dose, through inhibition of V-ATPase [98]. Farrag et al. demonstrated the chemopreventive efficacy of myrtenal against the bladder carcinogenesis of rats. The downregulation in the expressions of COX-2, NF-*κ*B, and STAT-3 correlated with the suppression of the levels of inflammatory cytokines of TNF-*α* and IL-6 and biomarkers of oxidative damage (MDA and NO). In addition, a significant increase in caspase-A3 activity and Bax/Bcl-2 ratio indicate that the anti-inflammatory effect and the induction of apoptosis contributed to this activity [99].

### 3.4. Monoterpenes That Induced Other Antitumor Mechanisms *In Vitro*

#### 3.4.1. *α*-Phellandrene

*α*-Phellandrene showed antitumor activity, which decreased the cell viability, promoted the cell cycle distribution, significantly increased reactive oxygen species levels, decreased mitochondrial membrane potential levels, increased the necrotic cell number, and increased NO production, LDH leakage, and ATP depletion on human liver cancer cells (J5) [100].

It was also seen that *α*-phellandrene upregulated DNA damage-associated genes and DNA fragmentation factor, cell cycle checkpoint genes, and apoptosis-associated genes. In addition, *α*-phellandrene has downregulated DNA damage-associated gene TATA box binding protein, D19Ertd652c (DNA segment), cell cycle-associated gene cyclin E2, apoptosis-associated gene growth arrest-specific 5, Gm5426 (ATP synthase), and death box polypeptide 33 [101].

In Lin et al. [102], mice were injected with mouse leukemia WEHI-3 cells and subsequently treated orally with or without *α*-PA. *α*-PA influences the murine WEHI-3 leukemia model *in vivo* by increasing the percentage of CD3 (T-cell marker), CD19 (B-cell marker), and MAC3 (macrophages) markers but reduced the percentage of CD11b (monocytes) cell surface markers. *α*-PA increased phagocytosis by macrophages and promoted natural killer cell activity. *α*-PA also increased B- and T-cell proliferation.

#### 3.4.2. Cymene

*p*-Cymene inhibits MMP-9 expression and increases TIMP-1 production besides inhibiting the ERK1/2 and p38 MAPK signal pathways on HT-1080 human fibrosarcoma cells, presenting a robust 87% inhibition of *in vitro* invasiveness [103]. *p*-Cymene is a natural antioxidant found in several plant species and is a constituent of fruits, wines, and spices, such as *Origanum vulgare* (oregano) and *Thymus vulgaris* (thyme). This compound has several pharmacological activities, in addition to an antinociceptive effect on cancer pain through inhibitory pathways and modulation of calcium currents [104–106].

#### 3.4.3. Rotundifolone

Rotundifolone, also known as piperitenone is a naturally occurring oxygenated monoterpene and represents one of the main components of the essential oil of many species of *Mentha* [107, 108]. Rotundifolone has recently been reported as presenting antioxidant and antiproliferative antitumor activities on U87MG glioblastoma cells with IC50 of 30 mg/L and alteration of PTEN/PI3K/AKT/NF-*κ*B signaling pathways [109].

The data described here may have implications for future research, possibly being used as a reference for the advancement in the mechanistic studies of these compounds, as well as in the preparation of synthetic derivatives or analogues with a better antitumor profile. Indeed, chemical modification in natural products is a current approach to improve drug actions against several diseases, including cancer [111].

## 4. Conclusions

The medicinal properties of essential oils have been evidenced through scientific investigations using experimental models. Considering that monoterpenes are commonly the main constituents of these oils, these natural products should contribute to pharmacological actions. The studies reported in this review confirm the antitumor properties of monoterpenes and their anticancer potential against various types of tumors, as demonstrated in *in vitro* and *in vivo* studies using various types of cancer cells and tumors in animal models. Since the last revision of this subject, several mechanisms of action of these compounds were elucidated, and deeper understanding of the use of theses monoterpenes in in *vivo* models was gained [14]. The main antitumor mechanism was through induction of apoptosis through several different pathways as inhibition of antiapoptotic proteins Bcl2 and BclXL or upregulation of cytochrome C release channel as BAX and BAK. Increase in ROS production and cell cycle impairment, mainly by disruption of cyclin D expression or CDK4 and its regulator p21, was also a common antitumor mechanism. Less common but not less interesting and important were autophagy induced by limonene and necroptosis by citronellol. Several tumor-related pathways were also regulated by these compounds inducing antiproliferative, death induction, decreased migration, or other phenotypes such as the oncogenic proteins JNK, Ras/MAPK, ERK1/2, p38, and PI3K; tumor suppressor proteins such as p53 and Chk1/2; and CDC25 and inflammation-related NF-*κ*B, TNF-*α*, IL1-*β*, COX2, and iNOS. The data described serve as a reference for the advancement in the mechanistic studies of these compounds and in the preparation of synthetic derivatives or analogues with a better antitumor profile.

## Figures and Tables

**Figure 1:** Chemical structure of antitumor monoterpenes found in essential oils.

**Table 1:** Essential oil monoterpenes with antitumor activity.

Compound	Antitumor activity and/or mechanism	Animal/cell line tested	IC50, % reference growth inhibition, dose, or selectivity	Reference
1,8-Cineole	Active (apoptosis and negligible necrotic effect)	A2780 (ovary cancer cells) and MRC5 (nontumorigenic human fetal lung fibroblasts)	0.26 *μ*g/mL and 10.50 *μ*g/mL (IC50), selective	[17]
	Active (cell cycle arrest and inhibition cell migration)	A549 (lung adenocarcinoma cells) and WI-38 (normal human embryonic lung fibroblasts)	8.30 *μ*g/mL, 5.84 *μ*g/mL, and >10 *μ*g/mL (IC50), selective	[19]
	Active (changes in mitochondrial membrane potential, apoptosis, and cell cycle arrest)	A431 (skin carcinoma) and HaCaT (human keratinocytes) cell lines	30 *μ*g/mL∗ (IC50), selective	[18]

*α*-Phellandrene	Active (altered gene expression)	WEHI-3 (mouse leukemia cells)	10 *μ*M^a^	[101]
	Active (reduced spleen weight, affected surface markers, increased macrophage phagocytosis, natural killer cell activity, and B- and T-cell proliferation)	Balb/c mice with mouse leukemia WEHI-3 cell injection	0, 25, and 50 mg/kg^b^	[102]
	Active (increase in reactive oxygen species, decrease in mitochondrial membrane potential levels, increase in the necrotic cell number, NO production, LDH leakage, and ATP depletion)	J5 (human liver tumor cells)	~30 *μ*M (IC50)	[100]

*α*-Pinene	Active (inhibition of cell growth; upregulation of Chk1 and Chk2 levels, and downregulation of Cyclin B, CDC25, and CDK1 levels; inhibition of tumor cell growth *in vitro* and *in vivo*; reduction of the average tumor size and the average tumor weight)	BEL-7402 (liver cancer cell) *in vitro* and balb nude mice	0.5-0.125 mg/L^a^; 2.67 mL/kg^b^; 79.3% (*in vitro* inhibitory rate) and 69.1%^c^;	[110]
			~70%^c^	
	Active (inhibition of the cell cycle and apoptosis)	PA-1 (cancer cells of the human ovary)	20 *μ*g/mL (IC50), 5-100 *μ*g/mL^a^	[33]
	NA (prevention of UVA-induced cytotoxicity)	HaCaT (human skin epidermal keratinocytes)	30 *μ*M^a^	[35]
	Active (apoptosis)	H460 and A549 non-small-cell lung cancer cell lines)	0.21 and 36.0 *μ*M (IC50), 2.5-20.0 *μ*M, and 0.0125-0.4 mg/mL^a^	[23]
	Active (cell cycle arrest, apoptosis, and oxidative stress)	HepG2 (liver cancer cells), MCF-7 (breast cancer cells), A549 (lung cancer cells), and PC-12 (neuroma cancer cells)	~100-1500 *μ*mol/L (IC50), 0-64 *μ*mol/L^a^	[34]

*α*-Thujone	Active (expression of CD107a, p-Akt, and p-ERK1/2)	HCT116 (human colon cancer cell line), SW620 (colon cancer cell line), and CD3AK (anti-CD3 antibody induced activated killer)	~0.01-0.15 *μ*mol/L (IC50), 0-37.5 *μ*mol/L^a^	[20]
	Active (apoptosis, inhibition of cell motility, oxidative stress, autophagy, and cell necrosis)	T98G and U87 (human glioblastoma multiforme cells) and C8-D1A (mouse astrocytes)	250 and 500 *μ*g/mL (IC50), 100-500 *μ*g/mL, and 660 *μ*M–3.2 mM^a^	[21]

Borneol	Active (“upper guiding drug”: guide luteolin in the ubiquitin-proteasome pathway and the ubiquitin-signal autophagic degradation)	Purification of 26S or 20S proteasome from pig red blood cells (RBCs) and HepG2 (hepatocellular carcinoma cells)	>1000 *μ*M (IC50), 100 and 500 *μ*M^a^	[37]
	Active (cell cycle arrest, production of reactive oxygen species, and DNA damage)	HepG2 (hepatocellular carcinoma cells) and L02 (normal liver cell lines)	>60 *μ*g/mL (IC50), 10-80 *μ*g/mL^a^, selective	[36]
	Active (cell cycle arrest, DNA damage, ROS production, enhanced dysfunction of MAPKs and PI3K/AKT pathways, and xenograft growth *in vivo*)	U251, U87 (human glioma cells), and HUVECs (human umbilical vein endothelial cells)	80 *μ*g/mL (IC50), 20-80%^c^	[38]
	Active (apoptosis, ROS production, and DNA damage)	U87 and U251 (human glioma cells) and HUVECs (human umbilical vein endothelial cells)	~40 *μ*g/mL (IC50), 5–80 *μ*M^a^	[39]

Bornyl acetate	Active (apoptosis, DNA fragmentation, and G2/M cell cycle arrest)	SGC-7901 (human gastric cancer cells)	~48 *μ*M (IC50), 0-96 *μ*M^a^	[22]

*β*-Pinene	Active (altered cell morphology, pyknotic nuclei, membrane blebs and cell shrinkage, and activated caspases)	SCC9 and SCC25 (human oral tongue cancer cells) and primary normal human gingival fibroblast	~67 *μ*g/mL (IC50), selective	[16]

Camphene	Active (apoptosis, loss of mitochondrial membrane potential, and inhibition of tumor growth)	B16F10-Nex2 (murine melanoma cell line), A2058 (melanoma cell line), SKBR-3 (breast cancer cell line), HeLa (cervical cancer cell line), HL-60 (human myeloid leukemia cell line), U87-MG (human glioblastoma cell line) *in vitro*, and C57Bl/6 mice	~27 and 110.1 *μ*g/mL (IC50), 0100 *μ*g/mL^a^, 10 mg/kg^b^, and 60%^c^	[42]

Carvacrol	Active (alteration in soluble factors)	HCT-116 and HT-29 (human colorectal carcinoma)	42 and 92 *μ*M (IC50), 25–200 *μ*M^a^	[50]
	Active (apoptosis and DNA damage)	AGS (human gastric adenocarcinomas), WS-1 (normal human fibroblast cells) *in vitro* and Wistar rats with oral gavage application of carvacrol	82.57 *μ*M (IC50), 0–600 *μ*M^a^, and 100 mg/kg^b^	[43]
	Active (ERK1/2-independent suppression of apoptosis and ERK1/2-dependent modulation of autophagy)	HeLa (human cervical cancer cell)	556 *μ*M (IC50), 550 *μ*M^a^	[49]
	Active (ROS production and apoptosis)	A549, PC-9 (human lung adenocarcinoma), BEAS-2B (normal bronchial epithelium cells) *in vitro*, and athymic nude mice with xenografting of A549 cells	100 *μ*g/mL (IC50), 25–150 *μ*g/mL^a^, 50 and 100 mg/kg^b^, 34.2%, and 62.1%^c^	[44]
	Active (downregulation of AXL expression, inhibited phosphorylation of AXL, and suppressed cell proliferation and migration)	A549 (human lung adenocarcinoma) and H460 (human lung cancer cells)	~100 and 300 *μ*M (IC50), 0-300 *μ*M^a^	[51]
	Active (apoptosis, reactive oxygen species generation, disruption in the mitochondrial membrane potential, and cell cycle arrest)	DU145 (human prostate cancer cells) and J774A.1 (normal mouse macrophage cells)	~50 and 100 *μ*M (IC50), 10-500 *μ*M^a^	[45]
	Active (inhibits proliferation and migration, cell cycle arrest, and apoptosis)	HCT116 and LoVo (human colon cancer cell lines)	530.2 and 544.4 *μ*mol/L (IC50), 200–900 *μ*mol/L^a^	[46]
	Active (suppressed the elevation of serum tumor marker enzymes, carcinoembryonic antigen, and *α*-feto protein and inhibited the cell proliferation)	Wistar albino rats with induction of hepatocarcinogenesis	15 mg/kg^b^	[52]
	NA (carvacrol has nonmutagenic and antioxidant features and decreased cell viability at high doses)	Human blood cells	0-200 mg/L^a^	[53]
	Active (apoptosis, collapse of mitochondrial membrane potential, generation of free radicals, and depletion of the intracellular antioxidant pool)	HL-60 (human acute promyelocytic leukemia cells) and Jurkat (T lymphoma cells)	50 *μ*M and 100 *μ*M (IC50), 0–200 *μ*M^a^	[47]
	Active (apoptosis, production of reactive oxygen species (ROS), mitochondrial membrane potential disruption, and prevented cell cycle in G0/G1)	PC-3 (prostate cancer cell line)	39.81 and 46.71 *μ*M (IC50), 10-500 *μ*M^a^	[48]

Carvone	Active (increased the total antioxidant capacity levels and increased the total oxidative stress levels)	Primary rat neuron cultures and rat brain NB cell line N2a	>400 mg/L (IC50), 10-400 mg/L^a^	[24]
	Active (synergistic anticancer action with doxorubicin)	MCF 7 (invasive breast ductal carcinoma), H9C2 (normal cardiomyocyte) *in vitro*, and BALB/c (Bagg albino) mice	14.22 *μ*M (IC50), 6.25 *μ*M-100 *μ*M^a^, and 75 and 150 mg/kg^b^	[27]
	Active (apoptosis)	Swiss albino mice with skin T tumorigenesis	20 mg/kg^b^, prevented tumor occurrence	[28]
	Active (inhibited the cell migration, apoptosis, cell cycle arrest, DNA damage, and ROS)	MCF 7 and MDA MB 231 (breast cancer cell lines) and MCF 10A (nontumorigenic epithelial cell line)	1.0 and 1.2 mM (IC50), 0-10 and 20 mM^a^	[25]
	Active (apoptosis, cell cycle arrest, and inhibited the cell invasion and expression of p-P38 protein)	KMS-5 (human myeloma cell line)	20 *μ*M (IC50), 0-100 *μ*M^a^	[26]

Citral	Active (arrested the cell migration, regulated several genes, and apoptosis)	AGS (human gastric adenocarcinomas) and MRC-5 (human lung normal cell lines)	~7.5 *μ*g/mL (IC50), 7.5-200 *μ*g/mL^a^	[54]
	Active (apoptosis)	MDA-MB-231, MDA-MB-468, and SKBR3 (breast cancer cell lines) *in vitro* and NOD/SCID female mice with MDA-MB-231 vector control or ALDH1A3 overexpression cells	100 mM^a^, 0.4 mg/kg^b^	[58]
	Active (impaired the clonogenic property of the cancer cells, suppressed lipogenesis and apoptosis)	PC-3 and PC3M (prostate cancer cells) and MRC-5 (human fetal lung fibroblast cell line)	10 and 12.5 *μ*g/mL (IC50), 0-100 *μ*g/mL^a^	[55]
	Active (inhibited the enzyme activity and the cell proliferation)	MCF-7 (breast cancer cell line), human embryonic (fetal) kidney, and HEK-293 cell lines	172 *μ*M (IC50), 0-400 *μ*M^a^, selective	[59]
	Active (apoptosis, reduced the mitochondrial membrane potential, elevated intracellular ROS level, and cell cycle arrest)	HCT116 and HT29 (colorectal cancer cell lines) and CCD841-CoN (normal colon cells)	52.63-181.21 *μ*g/mL (IC50), 3.12–200 *μ*M^a^	[56]
	Active (apoptosis)	Ramos (human Burkitt's lymphoma cell line) and PBMCs (normal human peripheral blood mononuclear cells)	77.19 *μ*M (IC50), 0–160 *μ*M^a^, selective	[57]
	Active (reduction the size and number of cells with ALDH+ activity of the tumors in 4T1-challenged BALB/c mice and delayed tumorigenicity)	BALB/c mice with 4T1 breast cancer cells	50 mg/kg^b^, 50%^c^	[60]

Citronellol	Active (upregulation of TNF-*α* pathway and increase in reactive oxygen species production)	NCI-H1299 (non-small-cell lung cancer) *in vitro* and in nude mice subcutaneous tumors	49.74 *μ*g/mL (IC50), selective, 50 mg/kg^b^, and 80%^c^	[61]
	Active (oxidative damage and modulation of the expression of apoptotic proteins)	MCF-7 and MDA-MB-231 (human mammary tumor cells)	35 and 80 *μ*M (IC50)	[62]

Cuminaldehyde	Active (inhibition of topoisomerase I and II activities)	COLO 205 (human colorectal adenocarcinoma cells) *in vitro* and in nude mice subcutaneous tumors	16.31 *μ*M (IC50), 20 mg/kg^b^, and 69.4%^c^	[93]
	Active (inhibition of telomerase, topoisomerase I and II activities)	A549 (human lung adenocarcinoma cells) *in vitro* and in nude mice subcutaneous tumors	18.33 *μ*M (IC50), 10 or 20 mg/kg^b^, and 50%^c^	[94]

*p*-Cymene	Active (inhibition of MMP-9 expression and increase of TIMP-1 production)	HT-1080 (human fibrosarcoma cells)	200-600 *μ*M^a^	[103]

Dehydroperillic acid	Active (inhibition of DNA synthesis)	A549 and HepG2 (human lung adenocarcinoma and hepatocellular carcinoma cells)	125 and >500 *μ*g/mL (IC50), SI = 400 and 100	[79]

Fenchone	Active (cell cycle arrest)	Ehrlich carcinoma cell line in the peritoneal cavities of mice	60 mg/kg^b^, ~90%^c^	[95]

Geraniol and geranyl acetate	Active (apoptosis, DNA damage, and cell cycle arrest)	Colo-205 (colon cancer cells)	20 and 30 *μ*M (IC50)	[63]

Geraniol	Active (downregulation of the activation of NF-*κ*B)	4NQO-induced tongue carcinogenesis in rats	ND	[64]
	Active (downregulation of E2F8)	PC-3 (prostate cancer cells)	1 mmol/L^a^	[65]
	Active (inhibition of the mevalonate pathway)	A549 (human lung adenocarcinoma cells) *in vitro* and in nude mice subcutaneous tumors	797.2 *μ*M (IC50), 50 and 75 mmol G/kg^b^, and ~83%^c^	[66]
	Active (apoptosis with involvement of the mitochondrial pathway)	Human Ishikawa endometrium cell line	~141 *μ*M (IC50)	[67]

Limonene	Active (apoptosis, cell cycle arrest, and suppression of cell migration and invasion)	T24 (human bladder cancer cell)	9 *μ*M (IC50)	[29]

Linalool	Active (inhibition of cell growth through cell cycle arrest)	A549 (human lung adenocarcinoma cells)	~1 and 1.7 mM (IC50), selective	[19]
	Active (cell cycle arrest, loss of mitochondrial membrane potential, and suppression of PI3K/AKT signaling pathway)	OECM 1 (human oral cancer cells)	10 *μ*M (IC50), SI = 6.5	[68]
	Active (oxidative stress)	HCT 116 (human colon cancer cell) *in vitro* and in SCID mice subcutaneous tumors	200 mg/kg^b^, 55%^c^	[69]
	Active (apoptosis and cell cycle arrest)	T-47D, SW 620, and HepG2 (breast, colorectal, and liver cancer cells)	224, 222, and 290 *μ*M (IC50)	[70]
	Active (cell cycle arrest and apoptosis through oxidative stress generation and modulation of Ras/MAPK and Akt/mTOR pathways)	HepG2 (hepatocellular carcinoma cells)	~1.1, 1.6, and 1.8 mM (IC50)	[71]
	Active (cell cycle arrest and apoptosis through CDKIs)	U937 and HeLa (leukemia and cervical cancer cells)	2.59 and 11.02 *μ*M (IC50)	[72]
	Active (oxidative stress)	Sarcoma-180 cells and sarcoma-180 solid tumor model in Swiss albino mice	~2 mM/L (IC50), 200 mg/kg^b^, and ~75%^c^	[73]

Myrtenal	Active (V-ATPase inhibition)	B16F0, B16F10, and SkMel-5 (murine and human melanoma cell lines) *in vitro* and in C57BL-6 mice subcutaneous and intravenously administration	5-200 *μ*M^a^, 15 mg/kg^b^, and ~50%^c^	[98]

Perillaldehyde 8,9-epoxide	Active (tumor growth inhibition)	Sarcoma 180-inoculated Swiss mice	100 and 200 mg/kg^b^, 38.4 and 58.7%^c^	[77]
	Active (apoptosis and necrosis)	OVCAR-8, HCT-116, SF-295, and HL-60 (human ovarian, colon, brain, and leukemia tumor cells)	0.64-1.75 *μ*L/mg (IC50)	[78]

Perillyl alcohol	Active (inhibition of HIF-1)	HeLa, SK-Hep1, and HCT116 (human cervical, hepatic, and colon cancer cells) *in vitro* and in nude mice subcutaneous tumors	5-200 *μ*M^a^, 100 mg/kg^b^, and 64.11%^c^	[75]
	Active (signaling mechanism mediated by Na/K-ATPase)	U251 and U87 (glioblastoma cells)	1.4 and 1.1 mM (IC50)	[74]
	Active (apoptosis)	AsPC-1, PANC-1, MIA PaCa-2, and BxPC-3 (pancreatic cancer cells) *in vitro* and in nude mice subcutaneous tumors	~100%^c^	[76]

Rotundifolone	Active (antioxidant and antiproliferative activities)	U87MG (glioblastoma cells)	30 mg/L (IC50)	[109]

Terpineol	Active (suppression of cell migration and induction of apoptosis and cell cycle arrest)	Hep-G2 (hepatocellular carcinoma cells) *in vitro* and in nude mice subcutaneous tumors	19.5 *μ*M (IC50), 20 mg/kg^b^, and ~75%^c^	[80]
	Active (apoptosis)	HT29, HCT116, COLO320, DLD1, AGS, COLO357, Panc-1, MIA-PACA, DU145, and CL-1 (human colorectal, gastric carcinoma, pancreas and prostate cancer cells) *in vitro* and in nude mice subcutaneous tumors	0.1% and 1%^b^, 40% and 70%^c^	[81]
	Active (inhibition of cell growth and induction of apoptosis)	BEL-7402 (human liver cancer cells)	0.32 mg/mL (IC50)	[82]

Thymoquinone	Active (apoptosis)	786-O (human renal carcinoma cells)	3.8–12.9 *μ*M (IC50)	[31]
Thymol and carvacrol	Active (apoptosis)	SKOV-3 (ovarian cancer cells)	258.38-322.50 *μ*M (IC50)	[83]

Thymol	Active (apoptosis)	PC-3, DU145, MDA-MB-231, and KLN205 (prostate, breast, and lung cancer cells)	208.36-799 *μ*M (IC50)	[84]
	Active (cell cycle arrest and mitochondria-mediated apoptosis)	T24, SW280, and J28 (bladder cancer cells)	90.1-130.5 *μ*M (IC50), selective	[85]
	Active (mitochondria-mediated apoptosis and tumor reduction)	Cal27, SCC4, and SCC9 (oral squamous cell carcinoma cells) *in vitro* and in nude mice subcutaneous tumors	300-550 *μ*M (IC50)	[86]
	Active (mitochondria-mediated apoptosis)	AGS (human gastric carcinoma cells)	100-400 *μ*M^a^	[87]
	None	HepG2 (hepatocarcinoma cells)	NA	[91]
	Active (mitochondria-mediated apoptosis)	A549 (non-small-cell lung cancer cells)	745 *μ*M (IC50)	[88]
	NA	Cultured human blood cells	10-200 mg/L^a^	[92]
	Active (mitochondria-mediated apoptosis)	HCT-116 (colorectal carcinoma cells)	100-200 *μ*g/mL^a^, selective	[89]
	Active (mitochondria-mediated apoptosis)	MCF-7 and MDA-MB231 (breast cancer cells)	47 and 56 *μ*g/mL (IC50)	[90]

Keys: Akt: protein kinase; ALDH: aldehyde dehydrogenase; ATP: adenosine triphosphate; AXL: receptor tyrosine kinase; CD107a: (or LAMP-1) lysosomal-associated membrane protein-1; CD3AK: anti-CD3 antibody induced activated killer; CDC25: cell division cycle 25 A; CDK1: cyclin-dependent kinase 1; CDKI: cyclin-dependent kinase inhibitor; Chk1: checkpoint kinase 1; Chk2: checkpoint kinase 2; DNA: deoxyribonucleic acid; E2F8: E2F transcription factor 8; ERK: extracellular signal-regulated kinase; IC50: half-maximal inhibitory concentration; LDH: lactate dehydrogenase; MAPK: mitogen-activated protein kinase; MMP-9: matrix metalloproteinase 9; mTOR: mammalian target of rapamycin; Na/K-ATPase: sodium-potassium pump; NF-kB: nuclear factor kappa B; p-Akt: phosphorylated protein kinase B; p-ERK: phosphorylated extracellular signal-regulated kinase; PI3K: phosphoinositide 3-kinase; p-P38: phospho-p38; ROS: reactive oxygen species; TIMP-1: tissue inhibitor of metalloprotease-1; TNF-*α*: tumor necrosis factor alpha; UVA: ultraviolet A; V-ATPase: vacuolar ATPase.

## Data Availability

The data in this review article were obtained from the PubMed database.

## Abbreviations

4NQO: 4-Nitroquinoline N-oxide
AKT: Protein kinase B (PKB), also known as AKT
ALDH+: Aldehyde dehydrogenase (ALDH)-positive
ALDH1A3: Aldehyde dehydrogenase 1A3
ATM: Ataxia telangiectasia mutated
AXL: AXL receptor tyrosine kinase
Bad: BCL2-associated agonist of cell death
BAK: Bcl-2 homologous antagonist/killer
BAX: Bcl-2-associated X protein
Bc-2: Serum biomarker
Bcl-2: Family of proteins that controls cell death
Bcl-xL: B-cell lymphoma-extra large
c-JUN: Protein encoded by the JUN gene
Ca2þ: Calcium ions
CD107a: Lysosome-associated membrane protein h-LAMP1
CD11b: Monocyte marker
CD19: B-cell marker
CD21: Cluster of differentiation 21
CD3: T-cell marker
CD3AK: Anti-CD3 antibody induced activated killer
CDC25: Dual-specificity phosphatase
CDK1: Cyclin-dependent kinase 1
CDK4: Cyclin-dependent kinase 4
Chk1: Checkpoint kinase 1
Chk2: Checkpoint kinase 2
CL-1: Androgen-independent prostate cancer cells
COX-2: Prostaglandin-endoperoxide synthase 2
CP: Cisplatin
Cyt-c: Cytochrome C
DOX: Doxorubicin
E2F8: E2F transcription factor 8
ERK: Extracellular signal-regulated kinase
Fas: Apoptosis-signaling receptor molecule
FDA: Food and Drug Administration
HIF-1: Hypoxia-inducible factor 1
HmgB1: High mobility group box 1
IC50: 50% inhibitory concentration
IFN-*γ*: Interferon *γ*
IL: Interleukin
iNOS: Inducible nitric oxide synthase
LDH: Lactate dehydrogenase
MAC3: Macrophage marker
MAPK: Mitogen-activated protein kinases
MARK4: Microtubule affinity regulating kinase 4
MEK: Mitogen-activated protein kinase kinase
MMP-9: Matrix metalloproteinase-9
mTOR: Mechanistic target of rapamycin
NA: Not applicable
NB: Natural borneol
ND: Not determined
NF-*κ*B: Nuclear factor-*κ*B
NO: Nitric oxide
p-Akt: Phosphorylated Akt
p-ERK1/2: Phospho-ERK1/2
p-JNK: Phospho-JNK
p-P38: Phospho-P38
p-PI3K: Phospho-PI3K
PARP: Poly(ADP-ribose)polymerase
PI3K: Phosphoinositide 3-kinases
ROS: Reactive oxygen species
TAC: Total antioxidant capacity
TIMP-1: TIMP metallopeptidase inhibitor 1
TNF-*α*: Tumor necrosis factor alpha
TOS: Total oxidative stress
ZDEVD: Caspase-3 inhibitor
ZVAD: Pancaspase inhibitor
*α*-PA: *α*-Phellandrene.

## References

[1] Sung H., Ferlay J., Siegel R. L. (2021). Global cancer statistics 2020: GLOBOCAN estimates of incidence and mortality worldwide for 36 cancers in 185 countries. *CA: a Cancer Journal for Clinicians*.

[2] Wang Y., Zhong J., Bai J. (2018). The application of natural products in cancer therapy by targeting apoptosis pathways. *Current Drug Metabolism*.

[3] Sharifi-Rad J., Ozleyen A., Boyunegmez Tumer T. (2019). Natural products and synthetic analogs as a source of antitumor drugs. *Biomolecules*.

[4] Yang Y., He P. Y., Zhang Y., Li N. (2020). Natural products targeting the mitochondria in cancers. *Molecules*.

[5] Abbas M. N., Kausar S., Cui H. (2020). Therapeutic potential of natural products in glioblastoma treatment: targeting key glioblastoma signaling pathways and epigenetic alterations. *Clinical & Translational Oncology*.

[6] Ren Y., Kinghorn A. D. (2019). Natural product triterpenoids and their semi-synthetic derivatives with potential anticancer activity. *Planta Medica*.

[7] Andrade M. A., Braga M. A., Cesar P. H. S. (2018). Anticancer properties of essential oils: an overview. *Current Cancer Drug Targets*.

[8] Gao X., Wei J., Hong L., Fan S., Hu G., Jia J. (2018). Comparative analysis of chemical composition, anti-inflammatory activity and antitumor activity in essential oils from *Siegesbeckia orientalis*, S. *glabrescens* and S. *pubescens* with an ITS sequence analysis. *Molecules*.

[9] Poma P., Labbozzetta M., McCubrey J. A. (2019). Antitumor mechanism of the essential oils from two succulent plants in multidrug resistance leukemia cell. *Pharmaceuticals (Basel)*.

[10] Wińska K., Mączka W., Łyczko J., Grabarczyk M., Czubaszek A., Szumny A. (2019). Essential oils as antimicrobial agents-myth or real alternative?. *Molecules*.

[11] Poma P., Labbozzetta M., Zito P. (2019). Essential oil composition of *Alluaudia procera* and in vitro biological activity on two drug-resistant models. *Molecules*.

[12] Britto A. C., de Oliveira A. C., Henriques R. M. (2012). *In vitro* and *in vivo* antitumor effects of the essential oil from the leaves of *Guatteria friesiana*. *Planta Medica*.

[13] Costa E. V., Menezes L. R., Rocha S. L. (2015). Antitumor properties of the leaf essential oil of *Zornia brasiliensis*. *Planta Medica*.

[14] Sobral M. V., Xavier A. L., Lima T. C., de Sousa D. P. (2014). Antitumor activity of monoterpenes found in essential oils. *The Scientific World Journal*.

[15] Bezerra D. P., Marinho Filho J. D., Alves A. P. (2009). Antitumor activity of the essential oil from the leaves of *Croton regelianus* and its component ascaridole. *Chemistry & Biodiversity*.

[16] Machado T. Q., Felisberto J. R. S., Guimarães E. F. (2022). Apoptotic effect of *β*-pinene on oral squamous cell carcinoma as one of the major compounds from essential oil of medicinal plant *Piper rivinoides* Kunth. *Natural Product Research*.

[17] Abdalla A. N., Shaheen U., Abdallah Q. M. A. (2020). Proapoptotic activity of *Achillea membranacea* essential oil and its major constituent 1,8-cineole against A2780 ovarian cancer cells. *Molecules*.

[18] Sampath S., Subramani S., Janardhanam S., Subramani P., Yuvaraj A., Chellan R. (2018). Bioactive compound 1,8-cineole selectively induces G2/M arrest in A431 cells through the upregulation of the p53 signaling pathway and molecular docking studies. *Phytomedicine*.

[19] Rodenak-Kladniew B., Castro M. A., Crespo R., Galle M., García de Bravo M. (2020). Anti-cancer mechanisms of linalool and 1,8-cineole in non-small cell lung cancer A549 cells. *Heliyon*.

[20] Zhou Y., Liu J. Q., Zhou Z. H. (2016). Enhancement of CD3AK cell proliferation and killing ability by *α*-thujone. *International Immunopharmacology*.

[21] Pudełek M., Catapano J., Kochanowski P. (2019). Therapeutic potential of monoterpene *α*-thujone, the main compound of *Thuja occidentalis* L. essential oil, against malignant glioblastoma multiforme cells in vitro. *Fitoterapia*.

[22] Li J., Wang S. X. (2016). Synergistic enhancement of the antitumor activity of 5-fluorouracil by bornyl acetate in SGC-7901 human gastric cancer cells and the determination of the underlying mechanism of action. *Journal of BUON*.

[23] Zhang Z., Guo S., Liu X., Gao X. (2015). Synergistic antitumor effect of *α*-pinene and *β*-pinene with paclitaxel against non-small-cell lung carcinoma (NSCLC). *Drug research*.

[24] Aydın E., Türkez H., Keleş M. S. (2015). Potential anticancer activity of carvone in N2a neuroblastoma cell line. *Toxicology and Industrial Health*.

[25] Patel P. B., Thakkar V. R. (2014). L-carvone induces p 53, caspase 3 mediated apoptosis and inhibits the migration of breast cancer cell lines. *Nutrition and Cancer*.

[26] Ding X., Chen H. (2018). Anticancer effects of carvone in myeloma cells is mediated through the inhibition of p 38 MAPK signalling pathway, apoptosis induction and inhibition of cell invasion. *Journal of BUON*.

[27] Abbas M. M., Kandil Y. İ., Abbas M. A. (2020). R-(-)-carvone attenuated doxorubicin induced cardiotoxicity *in vivo* and potentiated its anticancer toxicity *in vitro*. *Balkan Medical Journal*.

[28] Gopalakrishnan T., Ganapathy S., Veeran V., Namasivayam N. (2019). Preventive effect of D-carvone during DMBA induced mouse skin tumorigenesis by modulating xenobiotic metabolism and induction of apoptotic events. *Biomedicine & Pharmacotherapy*.

[29] Ye Z., Liang Z., Mi Q., Guo Y. (2020). Limonene terpenoid obstructs human bladder cancer cell (T24 cell line) growth by inducing cellular apoptosis, caspase activation, G2/M phase cell cycle arrest and stops cancer metastasis. *Journal of BUON*.

[30] Yu X., Lin H., Wang Y. (2018). D-limonene exhibits antitumor activity by inducing autophagy and apoptosis in lung cancer. *Oncotargets and Therapy*.

[31] Costa J. G., Keser V., Jackson C. (2020). A multiple endpoint approach reveals potential *in vitro* anticancer properties of thymoquinone in human renal carcinoma cells. *Food and Chemical Toxicology*.

[32] Samarghandian S., Azimi-Nezhad M., Farkhondeh T. (2019). Thymoquinone-induced antitumor and apoptosis in human lung adenocarcinoma cells. *Journal of Cellular Physiology*.

[33] Hou J., Zhang Y., Zhu Y. (2019). *α*-Pinene induces apoptotic cell death via caspase activation in human ovarian cancer cells. *Medical Science Monitor*.

[34] Xu Q., Li M., Yang M. (2018). *α*-Pinene regulates *miR-221* and induces G2/M phase cell cycle arrest in human hepatocellular carcinoma cells. *Bioscience Reports*.

[35] Karthikeyan R., Kanimozhi G., Prasad N. R., Agilan B., Ganesan M., Srithar G. (2018). Alpha pinene modulates UVA-induced oxidative stress, DNA damage and apoptosis in human skin epidermal keratinocytes. *Life Sciences*.

[36] Chen J., Li L., Su J., Chen T. (2015). Natural borneol enhances bisdemethoxycurcumin-induced cell cycle arrest in the G2/M phase through up-regulation of intracellular ROS in HepG2 cells. *Food & Function*.

[37] Chang T. L., Liou P. S., Cheng P. Y., Chang H. N., Tsai P. J. (2018). Borneol and luteolin from Chrysanthemum morifolium regulate ubiquitin signal degradation. *Journal of Agricultural and Food Chemistry*.

[38] Cao W. Q., Li Y., Hou Y. J. (2019). Enhanced anticancer efficiency of doxorubicin against human glioma by natural borneol through triggering ROS-mediated signal. *Biomedicine & Pharmacotherapy*.

[39] Cao W. Q., Zhai X. Q., Ma J. W. (2020). Natural borneol sensitizes human glioma cells to cisplatin-induced apoptosis by triggering ROS-mediated oxidative damage and regulation of MAPKs and PI3K/AKT pathway. *Pharmaceutical Biology*.

[40] Yang L., Liu H., Xia D., Wang S. (2020). Antioxidant properties of camphene-based thiosemicarbazones: experimental and theoretical evaluation. *Molecules*.

[41] Kim S., Choi Y., Choi S., Choi Y., Park T. (2014). Dietary camphene attenuates hepatic steatosis and insulin resistance in mice. *Obesity (Silver Spring)*.

[42] Girola N., Figueiredo C. R., Farias C. F. (2015). Camphene isolated from essential oil of Piper cernuum (Piperaceae) induces intrinsic apoptosis in melanoma cells and displays antitumor activity in vivo. *Biochemical and Biophysical Research Communications*.

[43] Günes-Bayir A., Kocyigit A., Güler E. M., Bilgin M. G., Ergün İ. S., Dadak A. (2018). Effects of carvacrol on human fibroblast (WS-1) and gastric adenocarcinoma (AGS) cells in vitro and on Wistar rats in vivo. *Molecular and Cellular Biochemistry*.

[44] Khan I., Bahuguna A., Kumar P., Bajpai V. K., Kang S. C. (2018). In vitro and in vivo antitumor potential of carvacrol nanoemulsion against human lung adenocarcinoma A549 cells via mitochondrial mediated apoptosis. *Scientific Reports*.

[45] Khan F., Khan I., Farooqui A., Ansari I. A. (2017). Carvacrol induces reactive oxygen species (ROS)-mediated apoptosis along with cell cycle arrest at G0/G1 in human prostate cancer cells. *Nutrition and Cancer*.

[46] Fan K., Li X., Cao Y. (2015). Carvacrol inhibits proliferation and induces apoptosis in human colon cancer cells. *Anti-Cancer Drugs*.

[47] Bhakkiyalakshmi E., Suganya N., Sireesh D. (2016). Carvacrol induces mitochondria-mediated apoptosis in HL-60 promyelocytic and Jurkat T lymphoma cells. *European Journal of Pharmacology*.

[48] Khan F., Singh V. K., Saeed M., Kausar M. A., Ansari I. A. (2019). Carvacrol induced program cell death and cell cycle arrest in androgen-independent human prostate cancer cells *via* inhibition of notch signaling. *Anti-Cancer Agents in Medicinal Chemistry*.

[49] Potočnjak I., Gobin I., Domitrović R. (2018). Carvacrol induces cytotoxicity in human cervical cancer cells but causes cisplatin resistance: involvement of MEK-ERK activation. *Phytotherapy Research*.

[50] Pakdemirli A., Karaca C., Sever T. (2020). Carvacrol alters soluble factors in HCT-116 and HT-29 cell lines. *Turkish Journal of Medical Sciences*.

[51] Jung C. Y., Kim S. Y., Lee C. (2018). Carvacrol targets AXL to inhibit cell proliferation and migration in non-small cell lung cancer cells. *Anticancer Research*.

[52] Subramaniyan J., Krishnan G., Balan R. (2014). Carvacrol modulates instability of xenobiotic metabolizing enzymes and downregulates the expressions of PCNA, MMP-2, and MMP-9 during diethylnitrosamine-induced hepatocarcinogenesis in rats. *Molecular and Cellular Biochemistry*.

[53] Türkez H., Aydın E. (2016). Investigation of cytotoxic, genotoxic and oxidative properties of carvacrol in human blood cells. *Toxicology and Industrial Health*.

[54] Balusamy S. R., Ramani S., Natarajan S., Kim Y. J., Perumalsamy H. (2019). Integrated transcriptome and *in vitro* analysis revealed anti-proliferative effect of citral in human stomach cancer through apoptosis. *Scientific Reports*.

[55] Balusamy S. R., Perumalsamy H., Veerappan K. (2020). Citral induced apoptosis through modulation of key genes involved in fatty acid biosynthesis in human prostate cancer cells: *in silico* and *in vitro* study. *BioMed research international*.

[56] Sheikh B. Y., Sarker M. M. R., Kamarudin M. N. A., Mohan G. (2017). Antiproliferative and apoptosis inducing effects of citral via p 53 and ROS-induced mitochondrial-mediated apoptosis in human colorectal HCT116 and HT29 cell lines. *Biomedicine & Pharmacotherapy*.

[57] Dangkong D., Limpanasithikul W. (2015). Effect of citral on the cytotoxicity of doxorubicin in human B-lymphoma cells. *Pharmaceutical Biology*.

[58] Thomas M. L., de Antueno R., Coyle K. M. (2016). Citral reduces breast tumor growth by inhibiting the cancer stem cell marker ALDH1A3. *Molecular Oncology*.

[59] Naz F., Khan F. I., Mohammad T. (2018). Investigation of molecular mechanism of recognition between citral and MARK4: a newer therapeutic approach to attenuate cancer cell progression. *International Journal of Biological Macromolecules*.

[60] Nigjeh S. E., Yeap S. K., Nordin N., Rahman H., Rosli R. (2019). In vivo anti-tumor effects of citral on 4T1 breast cancer cells via induction of apoptosis and downregulation of aldehyde dehydrogenase activity. *Molecules*.

[61] Yu W. N., Lai Y. J., Ma J. W. (2019). Citronellol induces necroptosis of human lung cancer cells *via* TNF-*α* pathway and reactive oxygen species accumulation. *In Vivo*.

[62] Rajendran J., Pachaiappan P., Thangarasu R. (2021). Citronellol, an acyclic monoterpene induces mitochondrial-mediated apoptosis through activation of proapoptotic factors in MCF-7 and MDA-MB-231 human mammary tumor cells. *Nutrition and Cancer*.

[63] Qi F., Yan Q., Zheng Z., Liu J., Chen Y., Zhang G. (2018). Geraniol and geranyl acetate induce potent anticancer effects in colon cancer Colo-205 cells by inducing apoptosis, DNA damage and cell cycle arrest. *Journal of BUON*.

[64] Madankumar A., Tamilarasi S., Premkumar T., Gopikrishnan M., Nagabhishek N., Devaki T. (2017). Geraniol attenuates 4NQO-induced tongue carcinogenesis through downregulating the activation of NF-*κ*B in rats. *Molecular and Cellular Biochemistry*.

[65] Lee S., Park Y. R., Kim S. H. (2016). Geraniol suppresses prostate cancer growth through down-regulation of E2F8. *Cancer Medicine*.

[66] Galle M., Crespo R., Kladniew B. R., Villegas S. M., Polo M., de Bravo M. G. (2014). Suppression by geraniol of the growth of A549 human lung adenocarcinoma cells and inhibition of the mevalonate pathway in culture and in vivo: potential use in cancer chemotherapy. *Nutrition and Cancer*.

[67] Kuzu B., Cüce G., Ayan İ. Ç. (2021). Evaluation of apoptosis pathway of geraniol on Ishikawa cells. *Nutrition and Cancer*.

[68] Pan W., Zhang G. (2019). Linalool monoterpene exerts potent antitumor effects in OECM 1 human oral cancer cells by inducing sub-G1 cell cycle arrest, loss of mitochondrial membrane potential and inhibition of PI3K/AKT biochemical pathway. *Journal of BUON*.

[69] Iwasaki K., Zheng Y. W., Murata S. (2016). Anticancer effect of linalool *via* cancer-specific hydroxyl radical generation in human colon cancer. *World Journal of Gastroenterology*.

[70] Chang M. Y., Shen Y. L. (2014). Linalool exhibits cytotoxic effects by activating antitumor immunity. *Molecules*.

[71] Rodenak-Kladniew B., Castro A., Stärkel P., De Saeger C., García de Bravo M., Crespo R. (2018). Linalool induces cell cycle arrest and apoptosis in HepG2 cells through oxidative stress generation and modulation of Ras/MAPK and Akt/mTOR pathways. *Life Sciences*.

[72] Chang M. Y., Shieh D. E., Chen C. C., Yeh C. S., Dong H. P. (2015). Linalool induces cell cycle arrest and apoptosis in leukemia cells and cervical cancer cells through CDKIs. *International Journal of Molecular Sciences*.

[73] Jana S., Patra K., Sarkar S. (2014). Antitumorigenic potential of linalool is accompanied by modulation of oxidative stress: an in vivo study in sarcoma-180 solid tumor model. *Nutrition and Cancer*.

[74] Garcia D. G., Castro-Faria-Neto H. C., Silva C. I. (2015). Na/K-ATPase as a target for anticancer drugs: studies with perillyl alcohol. *Molecular Cancer*.

[75] Ma J., Li J., Wang K. S. (2016). Perillyl alcohol efficiently scavenges activity of cellular ROS and inhibits the translational expression of hypoxia-inducible factor-1*α* via mTOR/4E-BP1 signaling pathways. *International Immunopharmacology*.

[76] Sarkar S., Azab B., Quinn B. A. (2014). Chemoprevention gene therapy (CGT) of pancreatic cancer using perillyl alcohol and a novel chimeric serotype cancer terminator virus. *Current Molecular Medicine*.

[77] Andrade L. N., Amaral R. G., Dória G. A. (2016). *In vivo* anti-tumor activity and toxicological evaluations of perillaldehyde 8,9-epoxide, a derivative of perillyl alcohol. *International Journal of Molecular Sciences*.

[78] Andrade L. N., Lima T. C., Amaral R. G. (2015). Evaluation of the cytotoxicity of structurally correlated p-menthane derivatives. *Molecules*.

[79] Oturanel C. E., Kıran İ., Özşen Ö., Çiftçi G. A., Atlı Ö. (2017). Cytotoxic, antiproliferative and apoptotic effects of perillyl alcohol and its biotransformation metabolite on A549 and HepG2 cancer cell lines. *Anti-Cancer Agents in Medicinal Chemistry*.

[80] Liu S., Zhao Y., Cui H. F., Cao C. Y., Zhang Y. B. (2016). 4-Terpineol exhibits potent in vitro and in vivo anticancer effects in Hep-G2 hepatocellular carcinoma cells by suppressing cell migration and inducing apoptosis and sub-G1 cell cycle arrest. *Journal of BUON*.

[81] Shapira S., Pleban S., Kazanov D., Tirosh P., Arber N. (2016). Terpinen-4-ol: a novel and promising therapeutic agent for human gastrointestinal cancers. *PLoS One*.

[82] Wu Z. L., Yin Z. Q., Du Y. H. (2014). *γ*-Terpineol inhibits cell growth and induces apoptosis in human liver cancer BEL-7402 cells *in vitro*. *International Journal of Clinical and Experimental Pathology*.

[83] Elbe H., Yigitturk G., Cavusoglu T., Baygar T., Ozgul Onal M., Ozturk F. (2020). Comparison of ultrastructural changes and the anticarcinogenic effects of thymol and carvacrol on ovarian cancer cells: which is more effective?. *Ultrastructural Pathology*.

[84] Elbe H., Yigitturk G., Cavusoglu T., Uyanikgil Y., Ozturk F. (2020). Apoptotic effects of thymol, a novel monoterpene phenol, on different types of cancer. *Bratislavské Lekárske Listy*.

[85] Li Y., Wen J. M., Du C. J. (2017). Thymol inhibits bladder cancer cell proliferation via inducing cell cycle arrest and apoptosis. *Biochemical and Biophysical Research Communications*.

[86] De La Chapa J. J., Singha P. K., Lee D. R., Gonzales C. B. (2018). Thymol inhibits oral squamous cell carcinoma growth via mitochondria-mediated apoptosis. *Journal of Oral Pathology & Medicine*.

[87] Kang S. H., Kim Y. S., Kim E. K. (2016). Anticancer effect of thymol on AGS human gastric carcinoma cells. *Journal of Microbiology and Biotechnology*.

[88] Balan D. J., Rajavel T., Das M., Sathya S., Jeyakumar M., Devi K. P. (2021). Thymol induces mitochondrial pathway-mediated apoptosis via ROS generation, macromolecular damage and SOD diminution in A549 cells. *Pharmacological Reports*.

[89] Chauhan A. K., Bahuguna A., Paul S., Kang S. C. (2018). Thymol elicits HCT-116 colorectal carcinoma cell death through induction of oxidative stress. *Anti-Cancer Agents in Medicinal Chemistry*.

[90] Jamali T., Kavoosi G., Safavi M., Ardestani S. K. (2018). *In-vitro* evaluation of apoptotic effect of OEO and thymol in 2D and 3D cell cultures and the study of their interaction mode with DNA. *Scientific Reports*.

[91] Shettigar N. B., Das S., Rao N. B., Rao S. B. (2015). Thymol, a monoterpene phenolic derivative of cymene, abrogates mercury-induced oxidative stress resultant cytotoxicity and genotoxicity in hepatocarcinoma cells. *Environmental Toxicology*.

[92] Aydin E., Türkez H. (2013). *In vitro* cytotoxicity, genotoxicity and antioxidant potentials of thymol on human blood cells. *Journal of Essential Oil Research*.

[93] Tsai K. D., Liu Y. H., Chen T. W. (2016). Cuminaldehyde from Cinnamomum verum induces cell death through targeting topoisomerase 1 and 2 in human colorectal adenocarcinoma COLO 205 cells. *Nutrients*.

[94] Chen T. W., Tsai K. D., Yang S. M. (2016). Discovery of a novel anti-cancer agent targeting both topoisomerase I & II as well as telomerase activities in human lung adenocarcinoma A549 cells in vitro and in vivo: Cinnamomum verum component cuminaldehyde. *Current Cancer Drug Targets*.

[95] Rolim T. L., Meireles D. R. P., Batista T. M. (2017). Toxicity and antitumor potential of *Mesosphaerum sidifolium* (Lamiaceae) oil and fenchone, its major component. *BMC Complementary and Alternative Medicine*.

[96] Pessoa M. L. S., Silva L. M. O., Araruna M. E. C. (2020). Antifungal activity and antidiarrheal activity via antimotility mechanisms of (-)-fenchone in experimental models. *World Journal of Gastroenterology*.

[97] Keskin I., Gunal Y., Ayla S. (2017). Effects of Foeniculum vulgare essential oil compounds, fenchone and limonene, on experimental wound healing. *Biotechnic & Histochemistry*.

[98] Martins B. X., Arruda R. F., Costa G. A. (2019). Myrtenal-induced V-ATPase inhibition - a toxicity mechanism behind tumor cell death and suppressed migration and invasion in melanoma. *Biochimica et Biophysica Acta - General Subjects*.

[99] Farrag M. A., Ezz M. K., Ibrahim N. K., Ahmed E. K. (2022). Chemopreventive potential of myrtenal against nitrosamine-initiated, radiation-promoted rat bladder carcinogenesis. *Nutrition and Cancer*.

[100] Hsieh S. L., Li Y. C., Chang W. C., Chung J. G., Hsieh L. C., Wu C. C. (2014). Induction of necrosis in human liver tumor cells by *α*-phellandrene. *Nutrition and Cancer*.

[101] Lin J. J., Yu C. C., Lu K. W. (2014). *α*-Phellandrene alters expression of genes associated with DNA damage, cell cycle, and apoptosis in murine leukemia WEHI-3 cells. *Anticancer Research*.

[102] Lin J. J., Lu K. W., Ma Y. S. (2014). Alpha-phellandrene, a natural active monoterpene, influences a murine WEHI-3 leukemia model in vivo by enhancing macrophague phagocytosis and natural killer cell activity. *In Vivo*.

[103] Li J., Liu C., Sato T. (2016). Novel antitumor invasive actions of p-cymene by decreasing MMP-9/TIMP-1 expression ratio in human fibrosarcoma HT-1080 cells. *Biological & Pharmaceutical Bulletin*.

[104] Cao X. L., Sparling M., Dabeka R. (2019). p-Cymene, a natural antioxidant, in Canadian total diet foods: occurrence and dietary exposures. *Journal of the Science of Food and Agriculture*.

[105] Santos W. B. R., Melo M. A. O., Alves R. S. (2019). p-Cymene attenuates cancer pain via inhibitory pathways and modulation of calcium currents. *Phytomedicine*.

[106] Formiga R. O., Alves Júnior E. B., Vasconcelos R. C. (2020). p-Cymene and rosmarinic acid ameliorate TNBS-induced intestinal inflammation upkeeping ZO-1 and MUC-2: role of antioxidant system and immunomodulation. *International Journal of Molecular Sciences*.

[107] de Sousa D. P., Lima T. C., Steverding D. (2016). Evaluation of antiparasitc activity of Mentha crispa essential oil, its major constituent rotundifolone and analogues against Trypanosoma brucei. *Planta Medica*.

[108] Di Sotto A., Di Giacomo S., Abete L. (2017). Genotoxicity assessment of piperitenone oxide: an *in vitro* and *in silico* evaluation. *Food and Chemical Toxicology*.

[109] Turkez H., Tozlu O. O., Lima T. C., de Brito A. E. M., de Sousa D. P. (2018). A comparative evaluation of the cytotoxic and antioxidant activity of *Mentha crispa* essential oil, its major constituent rotundifolone, and analogues on human glioblastoma. *Oxidative Medicine and Cellular Longevity*.

[110] Chen W., Liu Y., Li M. (2015). Anti-tumor effect of *α*-pinene on human hepatoma cell lines through inducing G2/M cell cycle arrest. *Journal of Pharmacological Sciences*.

[111] Yao H., Liu J., Xu S., Zhu Z., Xu J. (2017). The structural modification of natural products for novel drug discovery. *Expert opinion on drug discovery*.

